The article "Effect of Bimetal Element Doping on the Low-Temperature Activity of Manganese-Based Catalysts for NH3-SCR" was retracted in 2023. Reason: duplicate publication.

# Effect of Bimetal Element Doping on the Low-Temperature Activity of Manganese-Based Catalysts for NH_3_-SCR

**DOI:** 10.3389/fchem.2022.957051

**Published:** 2022-07-22

**Authors:** Haixia Li, Shuaibo Zhang, Anchao Zhang, Xinmin Zhang, Zhijun Sun, Changze Yang, Qifeng Zhu

**Affiliations:** School of Mechanical and Power Engineering, Henan Polytechnic University, Jiaozuo, China

**Keywords:** NH3-SCR, sulfur resistance, nitrogen oxide, metal modification, low temperature

## Abstract

A series of novel Mn_6_Zr_1-x_Co_x_ denitrification catalysts were prepared by the co-precipitation method. The effect of co-modification of MnO_x_ catalyst by zirconium and cobalt on the performance of NH_3_-SCR was studied by doping transition metal cobalt into the Mn_6_Zr_1_ catalyst. The ternary oxide catalyst Mn_6_Zr_0.3_Co_0.7_ can reach about 90% of NO_x_ conversion in a reaction temperature range of 100–275°C, and the best NO_x_ conversion can reach up to 99%. In addition, the sulfur resistance and water resistance of the Mn_6_Zr_0.3_Co_0.7_ catalyst were also tested. When the concentration of SO_2_ is 200ppm, the NO_x_ conversion of catalyst Mn_6_Zr_0.3_Co_0.7_ is still above 90%. 5 Vol% H_2_O has little effect on catalyst NO_x_ conversion. The results showed that the Mn_6_Zr_0.3_Co_0.7_ catalyst has excellent resistance to sulfur and water. Meanwhile, the catalyst was systematically characterized. The results showed that the addition of zirconium and cobalt changes the surface morphology of the catalyst. The specific surface area, pore size, and volume of the catalyst were increased, and the reduction temperature of the catalyst was decreased. In conclusion, the doping of zirconium and cobalt successfully improves the NH_3_-SCR activity of the catalyst.

## Highlights

- The ternary oxide catalyst Mn_6_Zr_0.3_Co_0.7_ catalyst was prepared by the co-precipitation method.
- The NO_x_ conversion of the Mn_6_Zr_0.3_Co_0.7_ catalyst is above 90% at 100–275°C.
- The Mn_6_Zr_0.3_Co_0.7_ catalyst has excellent resistance to H_2_O and SO_2_.
- The Mn_6_Zr_0.3_Co_0.7_ catalyst has a large specific surface area and pore diameter.
- The reaction mechanism of the Mn_6_Zr_0.3_Co_0.7_ catalyst was investigated.

## Introduction

With continuous exploitation and utilization of fossil fuels, serious pollution has been caused to the atmosphere, among which nitrogen oxide (NO_x_) is one of the most important pollutants. Therefore, the removal of NO_x_ is particularly important. At present, the most effective method for NO_x_ removal is selective catalytic reduction of NO_x_ with NH_3_ (NH_3_-SCR) (Zhang et al., 2015; Hu et al., 2017). In recent years, commercial SCR catalysts including V_2_O_5_/TiO_2_-WO_3_ and V_2_O_5_/TiO_2_-MoO_3_ had excellent deoxidation activity. However, because of the narrow operating temperature window, the activity of the catalyst is poor at low temperatures, and it can only work at high temperatures (350–450°C). In this way, the denitration device can only be installed at the front end of the desulfurization device, while the presence of SO_2_ in the flue gas can lead to V_2_O_5_/TiO_2_ catalyst inactivation (Shi et al., 2011; Hu et al., 2018). Therefore, the denitrification device can only be installed downstream of the desulfurization device, but this cannot meet the optimal reaction temperature of the V_2_O_5_/TiO_2_ catalyst (Jin et al., 2022). At the same time, the V_2_O_5_/TiO_2_ catalyst may also cause vanadium poisoning (Kwon et al., 2016; Hu et al., 2018). To sum up, it is particularly important to develop a kind of low-temperature and high-activity catalyst.

The article "Effect of Bimetal Element Doping on the Low-Temperature Activity of Manganese-Based Catalysts for NH3-SCR" was retracted in 2023. Reason: duplicate publication.

At present, the most widely studied catalysts are transition metal catalysts, zeolite catalysts, and rare earth metal catalysts. Among transition metal catalysts, manganese oxide (MnO_x_) catalysts have attracted much attention due to their excellent low-temperature SCR performance. However, the working temperature window of pure MnO_x_ catalyst is narrow, and when there is SO_2_ and H_2_O in the flue gas, the MnO_x_ catalyst will be inactivated, which seriously affects the denitration activity. Therefore, it is necessary to widen the temperature window of the MnO_x_ catalyst and improve the water and sulfur resistance. The Mn-Ce binary oxide catalyst prepared by the solvothermal method has abundant chemisorption oxygen and active sites and shows excellent low-temperature activity and significant sulfur resistance (Chen et al., 2021). Tang prepared Mn-Fe-Ce0.1 ternary oxide catalyst by the co-precipitation method, which has a large specific surface area and strong surface acidity, which is conducive to enhance the SCR denitration activity of the catalyst and improving the resistance to SO_2_ and H_2_O (Tang et al., 2020). In addition, MnAlO_x_ (Zhou et al., 2019), Fe‐Mn/Al_2_O_3_ (Wang et al., 2016), and Mn/TiWO_x_ (Chen et al., 2016a) have excellent SCR activity and water and sulfur resistance. Therefore, the introduction of one or more metal elements in the MnO_x_ catalyst can enhance the physicochemical properties of MnO_x_ catalyst so that the prepared catalyst has excellent denitrification performance.

Zirconium additives can improve the dispersity and activity of the catalyst and the sulfur resistance of the catalyst (Kantcheva et al., 2011). Ali synthesized the Cu_x_Ce_0.5-x_Zr_0.5_ oxide catalyst by the citric acid method, which showed excellent SCR activity, N_2_ selectivity, and water and sulfur resistance (Ali et al., 2017). Doped zirconium into the Cr_2_O_3_ catalyst by the co-precipitation method, which changed the surface performance of chromium oxide catalyst, improved the acid position of the CrZrO_x_ catalyst, the concentration of surface adsorbed oxygen O_a_ and Cr^6+^, and improved the SCR performance of the catalyst (Guo et al., 2021). In addition, Hu reported the influence of Co_3_O_4_ doping on NH_3_-SCR reaction in manganese-based catalyst, which greatly improved the redox capacity of the catalyst and proposed the reaction mechanism (Hu et al., 2015). Gao added cobalt to MnO_x_ through complexation esterification, and the catalyst showed good activity and improved the resistance of MnO_x_ to SO_2_ Gao et al. (2018). Zhang found that Mn_x_Co_3-x_O_4_ nanocages prepared by self-assembly have higher N_2_ selectivity, wider operating temperature range, and better SO_2_ tolerance compared with nanoparticles (Zhang et al., 2014). Therefore, the doping of zirconium and cobalt in manganese catalysts is of great research value.

The article "Effect of Bimetal Element Doping on the Low-Temperature Activity of Manganese-Based Catalysts for NH3-SCR" was retracted in 2023. Reason: duplicate publication.

In view of the reported effect of zirconium and cobalt on improving the catalytic activity and sulfur resistance of manganese-based catalysts, bimetal elements of zirconium and cobalt were added to the manganese-based catalysts simultaneously in the hope of preparing a more efficient denitration catalyst. In this study, a series of related Mn_6_Zr_1-x_Co_x_ catalysts were prepared by the co-precipitation method. The effects of cobalt-doped Mn_6_Zr_1_ bilayer oxides on the activity and resistance to SO_2_ and H_2_O were studied. In addition, the denitrification activity was tested in a fixed-bed reactor. The physicochemical properties of catalysts were investigated by conducting a series of related experiments and characterization, such as temperature-programmed technology, SEM, XRD, BET, XPS, H2-TPR, NH3-TPD, and *In Situ* DRIFTs.

## Experimental

### Materials

All samples were synthesized by the co-precipitation method with Mn(NO_3_)_2_·4H_2_O(99.0%, Macklin, Shanghai), Zr(NO_3_)_4_·5H_2_O(≥99.0%, Macklin, Shanghai), and Co(NO_3_)_2_·6H_2_O(≥99.0%, Macklin, Shanghai). NaOH (≥96.0%, Macklin, Shanghai) was used to regulate pH. (NH_4_)_2_CO_3_ (≥40.0%, MACKLIN, Shanghai) was used as the precipitator. In this study, none of the reagents used needs to be further purified.

### Catalyst Preparation

A series of Mn_6_Zr_1-x_Co_x_ catalysts were prepared by the co-precipitation method. Specifically, the corresponding precursor material was weighed, in which Mn: (Zr + Co) = 6:1, and the ratio of Zr: Co was 1:9, 3:7, 5:5, 7:3, and 9:1 (all ratios were molar ratios). Then, the mixed solution was put into five 300-ml beakers according to the proportion and marked with 1#, 2#, 3#, 4#, and 5#. Also, 100 ml of deionized water was added to each of the five beakers. The mixed solution was heated at 30°C in a water bath for 30 min and mixed with a magnetic stirrer at 500 r/min. 50 ml 0.5 mol L^−1^(NH_4_)_2_CO_3_ solution was gradually dropped into the abovementioned solution with full stirring for 2 h. Also, 0.5 mol·L^−1^NaOH solution was gradually added to the obtained solution to keep at pH = 9. The abovementioned solutions were aged at room temperature for 24 h, and then the supernatant was removed from the beaker and the sediment was collected. The sediment was washed with deionized water until neutral pH = 7. The washed sediments were dried at 105°C by using vacuum drying oven overnight to get the primary product. The primary products were calcined at 400°C for 3 h in a muffle furnace. Finally, solids were crushed and screened to 40–60 mesh to obtain the final experimental catalyst. Samples 1#, 2#, 3#, 4#, and 5# were Mn_6_Zr_0.1_Co_0.9_, Mn_6_Zr_0.3_Co_0.7_, Mn_6_Zr_0.5_Co_0.5_, Mn_6_Zr_0.7_Co_0.3,_ and Mn_6_Zr_0.9_Co_0.1_, respectively.

The article "Effect of Bimetal Element Doping on the Low-Temperature Activity of Manganese-Based Catalysts for NH3-SCR" was retracted in 2023. Reason: duplicate publication.

### Catalytic Performance Test

The activity of the catalyst was evaluated and detected by temperature-programmed technology, as shown in Figure 1. Each test used a catalyst (0.2 g,40–60 mesh) with a volume of about 0.5 ml, which was placed in a fixed-bed quartz reactor (diameter = 9 mm, length = 60 mm) for the NH_3_-SCR activity evaluation test. The reaction gas of NH_3_-SCR denitrification consists of 500 ppm NO, 500 ppm NH_3_, 5vol% O_2_, 100–200 ppm SO_2_ (when used), 5Vol% H_2_O (when used), and N_2_ as equilibrium gas. The total flow rate of the gas is 500 ml min^−1^, and the gas hourly space velocity (GHSV) was about 60,000 h^−1^. The reaction temperature was 100–300°C when the catalyst activity was tested. The concentrations of NO_x_ and O_2_ before and after the reaction were measured by a flue gas analyzer. The remaining unconverted gas is filtered with sodium hydroxide solution. Each temperature point was held for 30 min, and the data were recorded in a numerical stable state. NO_x_ conversion and N_2_ selectivity are calculated by the following equations, respectively:

$${\text{NO}}_{\text{x}}\text{ conversion}=\frac{{\left[{\text{NO}}_{\text{X}}\right]}_{\text{in}}-{\left[{\text{NO}}_{\text{X}}\right]}_{\text{out}}}{{\left[{\text{NO}}_{\text{X}}\right]}_{\text{in}}}\times 100\text{\%,}$$ (1)

$${\text{N}}_{2}\text{ selectivity}\left(\text{\%}\right)=\left(1-\frac{2{\left[{\text{N}}_{2}\text{O}\right]}_{\text{out}}+{\left[{\text{NO}}_{2}\right]}_{\text{out}}-2{\left[{\text{N}}_{2}\text{O}\right]}_{\text{in}}-{\left[{\text{NO}}_{2}\right]}_{\text{in}}}{{\left[{\text{NH}}_{3}\right]}_{\text{in}}+{\left[{\text{NO}}_{\text{X}}\right]}_{\text{in}}-{\left[{\text{NH}}_{3}\right]}_{\text{out}}-{\left[{\text{NO}}_{\text{X}}\right]}_{\text{out}}}\right)\times 100\text{\%}\text{.}$$ (2)

**FIGURE 1:** Catalytic activity evaluation device.

The article "Effect of Bimetal Element Doping on the Low-Temperature Activity of Manganese-Based Catalysts for NH3-SCR" was retracted in 2023. Reason: duplicate publication.

The SCR activity of the catalyst can also be quantitatively expressed by the first-order rate constant (k), which can be calculated by the formula of NO conversion (X) as follows (Gao et al., 2014; Jiang et al., 2020).

$$\text{k}=-\frac{{\text{F}}_{0}}{{\left[\text{NO}\right]}_{0}\text{W}}\text{ln}\left(1-\text{X}\right),$$ (3)

$$\text{Ink}=-\frac{{\text{E}}_{\text{a}}}{\text{RT}}+\text{lnA,}$$ (4)

where F_0_ is NO feeding rate; [NO]_0_ is NO concentration at the inlet; W is catalyst dosage; Ea is the apparent activation energy; T is the Kelvin temperature; R is the gas constant; A is the pre-exponential factor.

### Catalyst Characterization

The X-ray diffraction (XRD) test was carried out with Cu–Kα radiation (*λ* = 0.15418 nm) in a 40-kV and 40-mA X-ray tube by using a Bruker D8 Advance in Germany, and the scanning range is 10–80°. A scanning electron microscope (SEM), produced by Hitachi Company Japan, was used to analyze the morphology of the catalysts. Before the test, the sample is evenly smeared on the surface of the conductive adhesive and then sprayed with gold. The N_2_ adsorption–desorption isotherms of the catalysts were determined by using Quantachrome Instruments Quadrasorb Evo with high purity N_2_ as the adsorbent. Before each analysis, the catalysts were degassed in a vacuum at 300°C for 3 h, and isotherms were measured at liquid nitrogen N_2_ (−196°C). The speed is 6°/min. The XPS tester uses the Escalab 250XI spectrometer from Semer, Inc., operating under monochrome Al Kα radiation (1486.6 eV), 12 kV, and 15 mA ultra-high vacuum, and all binding energies were calibrated by C1s peak at 284.4 eV. Temperature programmed reduction of H_2_ (H_2_-TPR) and temperature-programmed desorption of NH_3_ (NH_3_-TPD) were performed on the Mac AutoChem II 2920 instrument (United States). The former was pretreated in 300°C argon at a flow rate of 20 ml/min for 1h and cooled to room temperature. The gas was converted into a mixture of 5Vol % H_2_-N_2_ at a flow rate of 30 ml/min. After a straight baseline, the catalyst was heated from room temperature to 800°C at a rate of 10°C/min. The latter was pretreated in 300°C argon at a flow rate of 20 ml/min for 1 h and cooled to room temperature. The samples were then exposed to a mixture of 5 vol% NH_3_-N_2_ for 1 h and then purified with high-purity He at a flow rate of 20 ml/min to remove the physically adsorbed NH_3_. After the baseline was stabilized, the sample was heated from room temperature to 800°C at a rate of 10°C/min. The *in situ* Diffuse Reflectance Infrared Transform Spectroscopy (*in situ* DRIFTS) experiments were applied on a Thermo fisher Nicolet iS50 FTIR spectrometer to characterize the desorption of NO and NH_3_ on catalytic materials.

The article "Effect of Bimetal Element Doping on the Low-Temperature Activity of Manganese-Based Catalysts for NH3-SCR" was retracted in 2023. Reason: duplicate publication.

## Evaluation of Catalyst Activity

### Catalytic Activity for NH_3_-SCR

All samples were tested for the catalytic performance of NH_3_-SCR and the results are shown in Figure 2A. The NO_x_ conversion of all catalysts increased first and then decreased with the increase of reaction temperature. When the reaction temperature is 125–250°C, the NO_x_ conversion of the Mn_6_Zr_1_ catalyst is more than 90%, showing excellent catalytic activity. The effect of Co/Zr ratios on NH_3_-SCR performance of Mn_6_Zr_1-x_Co_x_ catalysts is shown in Figure 2A. It is worth noting that the NOx conversion first declines and then enhances with the increase of Co ratio. Among these catalysts, the Mn_6_Zr_0.3_Co_0.7_ catalyst exhibits optimal NH_3_-SCR activity with the NO_x_ conversion being above 90% in the range of 100–275°C and 99% in the range of 150–225°C. However, the Mn_6_Zr_0.5_Co_0.5_ catalyst shows the worst NH_3_-SCR activity. These findings indicate that the high same Co/Zr content does not improve the catalytic performance of NO_x_ conversion. This may be because the combination of zirconium and cobalt can change the physical and chemical properties of the catalyst surface, thus affecting the adsorption, redox, and surface reaction of active molecules on the catalyst surface. Meanwhile, the N_2_ selectivity of all catalysts was tested, as shown in Figure 2B, The selectivity of N_2_ decreases with the increase of reaction temperature, which may be related to the formation of N_2_O on the catalyst. When the Mn_6_Zr_1_ catalyst is doped with cobalt, the selectivity of N_2_ is obviously improved. At 100–200°C, the N_2_ selectivity of the Mn_6_Zr_0.3_Co_0.7_ catalyst is above 80%, and the optimum N_2_ selectivity is 96%. In conclusion, cobalt doping in the Mn_6_Zr_1_ catalyst significantly enhances its catalytic activity, widens the temperature window, and improves the selectivity of N_2_.

**FIGURE 2:** NO_x_ conversion **(A)** and N_2_ selectivity **(B)** over Mn_6_Zr_1-x_Co_x_ catalysts.

### SO_2_ and H_2_O Tolerance Resistance of Catalyst

In order to simulate the flue gas atmosphere under the actual conditions, the denitration efficiency of the catalyst was tested under the conditions containing SO_2_ or H_2_O, which were all measured at the optimum reaction temperature. The NO_x_ conversion in the SO_2_ atmosphere is shown in Figure 3A. The Mn_6_Zr_0.3_Co_0.7_ catalyst has significantly higher sulfur resistance than the Mn_6_Zr_1_ catalyst. The NO_x_ conversion of the Mn_6_Zr_0.3_Co_0.7_ catalyst stabilized at 95% after 4 h when 100 ppm SO_2_ was injected into the simulated flue gas. The NO_x_ conversion of the Mn_6_Zr_0.3_Co_0.7_ catalyst remains above 90% when 200 ppm SO_2_ is added. The results indicated that cobalt doping in the Mn_6_Zr_1_ catalyst significantly improved its resistance to sulfur. The main reason may be that cobalt doping into the Mn_6_Zr_1_ catalyst increases the active sites on the catalyst surface and changes the physicochemical properties and redox performance of the catalyst. In addition, the NO_x_ conversion of two kinds of catalyst did not recover to the initial NO_x_ conversion after the SO_2_ was turned off, mainly because SO_2_ and NH_3_ reaction formation sulfate or metal oxides are difficult to decompose under low-temperature, which covers some active sites on the catalyst and acid sites, and the activity cannot recover to the original SCR catalysts (Jia et al., 2018). At the same time, the water tolerance test of the catalyst was measured under the condition of 5Vol% H_2_O, and the results are shown in Figure 3B. The results showed that when 5Vol% H_2_O is added to the simulated gas, the NO_x_ conversion of the two catalysts decreases and the conversion of the catalysts is basically stable after 8 h. The conversion of the Mn_6_Zr_0.3_Co_0.7_ catalyst is stable at 95% and that of Mn_6_Zr_1_ catalyst is stable at 92%. The Mn_6_Zr_0.3_Co_0.7_ catalyst showed the best water resistance, indicating that the doping of cobalt also improved the water resistance of the Mn_6_Zr_1_ catalyst. The NO_x_ conversion of the Mn_6_Zr_0.3_Co_0.7_ catalyst recovered up to 99% of the initial value after the water vapor was turned off, indicating that the catalyst was reversible.

The article "Effect of Bimetal Element Doping on the Low-Temperature Activity of Manganese-Based Catalysts for NH3-SCR" was retracted in 2023. Reason: duplicate publication.

**FIGURE 3:** SO_2_ resistance **(A)** and H_2_O resistance **(B)** of Mn_6_Zr_1_ and Mn_6_Zr_0.3_Co_0.7_ catalysts.

## Characterization Analysis of Catalysts

### Crystal Structure Analysis

In order to understand the crystal structure of the catalysts, all the catalysts were characterized by XRD, and the results are shown in Figure 4. It can be seen that MnO_2_(PDF#12-0141) and Mn_3_O_4_(PDF#04-0732) species exist on the Mn_6_Zr_1_ catalyst. The diffraction peaks of Mn_6_Zr_1-x_Co_x_ series catalysts decrease gradually with the decrease of doping cobalt content x. This indicates that MnO_x_ species are highly dispersed and form a microcrystalline structure on the Mn_6_Zr_1-x_Co_x_ catalyst, which contributes to the improvement of catalyst activity (Gong et al., 2020). In addition, when 2Ɵ = 55°, there is a wide diffraction peak, which can be understood as the mixed oxide of MnO_2_ and Mn_3_O_4_. The wide peak structure is conducive to the adsorption, desorption, and redox reaction on the catalyst surface (Tang et al., 2007). It is worth noting that the phases of ZrO_2_ and CoO_x_ were not detected on all the catalysts, indicating that the phases related to them are likely to be introduced into the lattice of MnO_x_ to form a solid solution (Azalim et al., 2011).

**FIGURE 4:** XRD patterns of Mn_6_Zr_1-x_Co_x_ catalysts.

### Crystal Morphology Analysis

Figure 5 shows the SEM morphology of CoO_x_, Mn_6_Zr_1,_ and Mn_6_Zr_0.3_Co_0.7_ catalysts. As shown in Figure 5A, the morphology of CoO_x_ is an irregular block structure. As shown in Figure 5B,C the Mn_6_Zr_1_ catalyst present a cubic structure. It was found that the surface morphology of the original catalyst changed significantly after doping cobalt. As can be seen from Figures 5D,E, the morphology of the Mn_6_Zr_0.3_Co_0.7_ catalyst changes into a spherical structure with a diameter of 26 μm. In addition, Figure 5F clearly shows that the surface of Mn_6_Zr_0.3_Co_0.7_ catalyst forms a villous structure of about 1 μm. Such villi increase the specific surface area of the catalyst and the active sites on the surface. In the SCR denitration process, the reaction molecules can be captured better, thus promoting the denitration activity of the catalyst.

**FIGURE 5:** SEM image of **(A)** CoO_x_, **(B)** Mn_6_Zr_1_, and **(C)** Mn_6_Zr_0.3_Co_0.7_.

### Specific Surface Area and Pore Structure Analysis

Figure 6 shows the N_2_ adsorption isotherms and pore size distribution of the three catalysts of Mn_6_Zr_1_, CoO_x_, and Mn_6_Zr_0.3_Co_0.7_ at liquid nitrogen temperature. The specific surface area, pore volume, and pore diameter of the three catalysts are shown in Table 1. In Figure 6A, the shapes of all isotherms can be regarded as type IV isotherms, which are characteristic of mesoporous materials (Jia et al., 2017). All the isotherms of the samples have lagged rings which can be attributed to type H3. When P/P_0_ relative pressure is low, N_2_ adsorption increases sharply, indicating the presence of narrow micropores in the catalyst (Huang et al., 2021). Figure 6B shows the pore size distribution of the catalyst. The results showed that the peak of the three catalysts at 2 nm belongs to micropore aggregation, and the wide peak at 3–7 nm belongs to mesoporous distribution. It shows that the samples are mainly mesoporous, supplemented by microporous. There are many intermediate holes in the catalyst, which are conducive to the removal of NO_x_, thus showing good catalytic activity. Table1 shows that the specific surface area, pore volume, and pore size of the Mn_6_Zr_0.3_Co_0.7_ catalyst are increased to 156 m^2^/g, 0.29 cm^3^/g, and 3.7 nm, respectively, after the addition of cobalt. The results are consistent with SEM analysis of the Mn_6_Zr_0.3_Co_0.7_ catalyst. The increase of specific surface area is conducive to the dispersion of the active substance and the contact between the active site and the reactants, and the larger pore size can promote the rapid passage of the reactive gas, thus improving the NH_3_-SCR activity of the catalyst (Zhai et al., 2021).

The article "Effect of Bimetal Element Doping on the Low-Temperature Activity of Manganese-Based Catalysts for NH3-SCR" was retracted in 2023. Reason: duplicate publication.

**FIGURE 6:** **(A)** N_2_ adsorption isotherms and **(B)** pore size distributions of Mn_6_Zr_1_, Mn_6_Zr_0.3_Co_0.7,_ and CoO_x_.

**TABLE 1:** Surface areas, pore-volume, and average pore diameter of the samples.

Samples	Surface area (m^2^/g)	Pore volume (cm^3^/g)	Average pore diameter (nm)
Mn_6_Zr_1_	153	0.28	2.5
CoO_x_	109.3	0.28	6.7
Mn_6_Zr_0.3_Co_0.7_	155.6	0.29	3.7

### Analysis of Surface Element Composition

The surface elemental states of Mn_6_Zr_1_ and Mn_6_Zr_0.3_Co_0.7_ catalysts were characterized by XPS technology. The XPS analysis results are shown in Figure 7 and Table 2. The XPS spectra of Mn 2p showed two main peaks including Mn2p_3/2_ and Mn2p_1/2_. Through peak fitting deconvolution, the three characteristic peaks of Mn^4+^, Mn^3+^, and Mn^2+^ in Mn2P_3/2_ on the Mn_6_Zr_1_ catalyst are 643.1, 641.7,, and 640.6 eV, respectively. Mn2p_3/2_ is divided into the three characteristic peaks of 643.2, 641.9,, and 640.7 eV on the Mn_6_Zr_0.3_Co_0.7_ catalyst corresponding to the binding energies of Mn^4+^, Mn^3+^, and Mn^2+^, respectively (Chen et al., 2020; Pan et al., 2020). As can be seen from Table 2, when the Co element is doped in the Mn_6_Zr_1_ catalyst, the Mn^4+^/Mn ratio in the Mn_6_Zr_0.3_Co_0.7_ catalyst is significantly higher than that obtained by Mn_6_Zr_1_. One possible reason is the interaction of cobalt and zirconium with manganese oxides. The ratio of Mn^4+^/Mn in the Mn_6_Zr_0.3_Co_0.7_ catalyst is larger than that of Mn^3+^/Mn, indicating that Mn^4+^ is dominant. In addition, the Mn^4+^ has the strongest catalytic activity in the NH_3_-SCR reaction. This is one of the important reasons for the excellent activity of the Mn_6_Zr_0.3_Co_0.7_ catalyst (Chen et al., 2016b).

**FIGURE 7:** XPS spectra of **(A)** Mn2p **(B)** O1s, **(C)** Zr3d, and **(D)** Co2p of the Mn_6_Zr_1_ and Mn_6_Zr_0.3_Co_0.7_.

**TABLE 2:** XPS test results of Mn_6_Zr_1_ and Mn_6_Zr_0.3_Co_0.7_ catalysts.

Catalysts	Mn 2p		O 1s	Co 2p	
	Mn^3+^/Mn	Mn^4+^/Mn	O_α_/(O_α_+O_β_)	Co^3+^/Co	Co3+/Co2+
Mn_6_Zr_1_	34.32%	46.54%	47.94%	0	0
Mn_6_Zr_0.3_Co_0.7_	31.04%	50.13%	48.16%	57%	133%

Figure 7B shows the XPS spectra of O1s of the two catalysts. The O1s peaks of both catalysts were composed of two fitting peaks of 529.5–529.8 eV and 531.1–531.4 eV, respectively. The former is attributed to lattice oxygen, denoted as O_β_; The latter is attributed to adsorbed oxygen, denoted as O_α_ (Boningari et al., 2015). Table 2 shows that the O_α_/(O_α_+O_β_) value of the Mn_6_Zr_0.3_Co_0.7_ catalyst is 48.16%, which is higher than that of Mn_6_Zr_1_ (47.97%). It can be seen that the adsorbed oxygen on the surface of Mn_6_Zr_1_ is more abundant. Since the mobility of chemisorbed oxygen is higher than that of lattice oxygen, chemisorbed oxygen is generally more active than lattice oxygen (Fan et al., 2018). Therefore, a higher O_α_/(O_α_+O_β_) ratio is favorable for low-temperature NH_3_-SCR reaction and capable of promoting the oxidation of NO to NO_2_, thus accelerating the “Fast SCR” reaction (Zhang et al., 2018; Wu et al., 2021).

The article "Effect of Bimetal Element Doping on the Low-Temperature Activity of Manganese-Based Catalysts for NH3-SCR" was retracted in 2023. Reason: duplicate publication.

Figure 7C is the XPS spectrum of Zr3d. The binding energies of Mn_6_Zr_1_ and Mn_6_Zr_0.3_Co_0.7_ catalysts at Zr3d_5/2_ are 181.9 and 181.7 eV, respectively. The binding energy of Zr3d_5/2_ on pure ZrO_2_ is 182.1 eV (Fang et al., 2018). The binding energy Mn_6_Zr_0.3_Co_0.7_ is significantly lower than that of the two other catalysts. A lower binding energy means more active elements, which will ultimately improve the catalytic reaction (Fang et al., 2017).

The XPS spectrum of Co2p is shown in Figure 7D. It can be seen that Co2p3/2 is fitted into three peaks. The peak at 780.3eV can be attributed to Co3+. The peak at 781.8 eV can be attributed to Co2+, and the other peak belongs to the satellite peak with a peak of 786.5 eV (Wang et al., 2019). According to the literature, Co3+ plays an important role in NH3-SCR reaction. More Co3+ species on the catalyst surface, the better the redox performance of the catalyst (Meng et al., 2013). As can be seen from Table 2, the values of Co3+/Co and Co3+/Co2+ indicate that there are a large number of Co3+ species on the surface of the Mn_6_Zr_0.3_Co_0.7_ catalyst, and Co3+ occupies a dominant position, which well proves the reason for the excellent catalyst activity.

### Temperature Programming Testing

The surface acidity of the catalyst is also very important in NH_3_-SCR reactions. The surface acidity of the catalyst was investigated by using NH_3_-TPD. As can be seen from Figure 8A, the desorption peaks of the two catalysts at around 100°C may be due to the physical adsorption of NH_3_ at the weak acid site, and part of NH_4_^+^ ions are adsorbed by the Brønsted acid site. The desorption peaks at 239 and 242°C are the chemical adsorption of NH_3_ at the weak acid site (Liu et al., 2012; Jia et al., 2017). There is a desorption peak for catalyst Mn_6_Zr_1_ at 490°C and a desorption peak for catalyst Mn_6_Zr_0.3_Co_0.7_ at 522°C, both of which can be attributed to the adsorption of NH_3_ at the Lewis acid site, but the former belongs to the medium acid site and the latter belongs to the strong acid site (Fang et al., 2013). As is known to all, the desorption peak area of the catalyst represents the amount of catalyst acid. By integrating the NH_3_-TPD curve, the number of acid centers on the surface of Mn_6_Zr_0.3_Co_0.7_ and Mn_6_Zr_1_ catalysts can be estimated. It can be seen from the integral region of Figure 8A that the acid content of the Mn_6_Zr_0.3_Co_0.7_ catalyst is 17.3 μmol g^−1^, which is significantly higher than that of the Mn_6_Zr_1_ catalyst 13.64 μmol g^−1^. The results showed that the addition of cobalt not only enhanced the acidity of the catalyst surface but also increased the amount of acid, which was conducive to the adsorption of NH_3_ and promoted the SCR reaction.

The article "Effect of Bimetal Element Doping on the Low-Temperature Activity of Manganese-Based Catalysts for NH3-SCR" was retracted in 2023. Reason: duplicate publication.

**FIGURE 8:** **(A)** NH_3_-TPD profiles of Mn_6_Zr_1_ and Mn_6_Zr_0.3_Co_0.7_ catalysts and **(B)**H_2_-TPR profiles of Mn_6_Zr_1_ and Mn_6_Zr_0.3_Co_0.7_ catalysts.

H_2_-TPR was used to evaluate the redox performance of each catalyst and the interaction between the support and the active component. The redox capacity of the sample depended on the initial reduction temperature. In Figure 8B, both Mn_6_Zr_1_ and Mn_6_Zr_0.3_Co_0.7_ catalysts have two reduction peaks. Studies had showed that all manganese-based catalysts follow MnO_2_→Mn_3_O_4_→Mn_2_O_3_→MnO (Thirupathi and Smirniotis, 2011; France et al., 2017). Both catalysts show reduction peaks at 200–300°C and 300–500°C. The former can be attributed to the reduction of Mn^4+^→Mn^3+^ and Co^3+^→Co^2+^, while the latter can be attributed to the reduction of Mn^3+^→Mn^2+^ and Co^2+^→Co (Jiang and Song, 2013; Sun et al., 2018). The peak of the Mn_6_Zr_0.3_Co_0.7_ catalyst in the temperature range of 500–700°C can be attributed to the reduction of CoO (Lamonier et al., 2007). In addition, the reduction peak temperature of the Mn_6_Zr_0.3_Co_0.7_ catalyst is significantly lower than that of the Mn_6_Zr_1_ catalyst, which may be due to the formation of more surface oxygen vacancies in SCR reaction, which is conducive to the enhancement of oxygen fluidity or activation of reactants (Boningari et al., 2015). This indicates that the doping of cobalt enhances the redox capacity of the catalyst, which well-explains the reason why the Mn_6_Zr_0.3_Co_0.7_ catalyst has a good low-temperature denitration activity.

The article "Effect of Bimetal Element Doping on the Low-Temperature Activity of Manganese-Based Catalysts for NH3-SCR" was retracted in 2023. Reason: duplicate publication.

### *In situ* DRIFT Analysis

The adsorption reaction of NH_3_ and NO_x_ on the Mn_6_Zr_0.3_Co_0.7_ catalyst is the key to the SCR process. Therefore, *in situ* DRIFT spectra were carried out, and the results are shown in Figure 9. At 200°C, the Mn_6_Zr_0.3_Co_0.7_ sample was pre-adsorbed with NH_3_ for 60min and then purged with N_2_ for 30 min. After removing the physically adsorbed ammonia, the Mn_6_Zr_0.3_Co_0.7_ catalyst was exposed to the mixture of NO + O_2_. The peaks at 1622 cm^−1^ and 1170 cm^−1^ were observed after NH_3_ adsorption, which was due to the coordination state of NH_3_ at the Lewis acid site on the catalyst surface (Han et al., 2019; Xiong et al., 2020). The characteristic peaks at 1450 cm^−1^ and 1420 cm^−1^ are attributed to the stretching vibration of NH_4_^+^ at the Brønsted acid sites (Zhang et al., 2021; Ge et al., 2022). Lewis and Brønsted acid sites coexist on the Mn_6_Zr_0.3_Co_0.7_ catalyst surface. In addition, a characteristic peak of coordination NH_3_ appeared at 1215 cm^−1^ (Han et al., 2019). The band at 1070 cm^−1^ belongs to the active intermediate species NH_2_. With the introduction of NO + O_2_, the intensity of characteristic peaks of NH_4_^+^, coordination NH_3_, and amide (-NH_2_) gradually decreased and disappeared rapidly. Bridging nitrates (1629 cm^−1^, 1599 cm^−1^, and 1230 cm^−1^), bridged bidentate nitrate (1270 cm^−1^), and nitrates (998 cm^−1^) were formed (Han et al., 2019; Gong et al., 2020). All coordination NH_3_, NH_4_^+^, and -NH_2_ are involved in the reaction. The removal of NO by NH_3_-SCR on the Mn_6_Zr_0.3_Co_0.7_ catalyst follows L-H and E-R mechanisms according to the change of the characteristic peak of the *in situ* drift spectrum.

**FIGURE 9:** *In situ* DRIFT spectra of NO + O_2_ reaction with pre-adsorbed NH_3_ over the Mn_6_Zr_0.3_Co_0.7_ catalyst at 200°C.

### Kinetic Analysis

The SCR activity differences of Mn_6_Zr_1_ and Mn_6_Zr_0.3_Co_0.7_ catalysts were further investigated by kinetic experiments. According to the Arrhenius formula, the apparent activation energy Ea of NO_x_ conversion can be obtained by the slope of the Lnk curve along with 1/T, as shown in Figure 10. It can be seen that the apparent activation energy Ea of Mn_6_Zr_1_ and Mn_6_Zr_0.3_Co_0.7_ catalysts is 22.53 kJ/mol and 5.41 kJ/mol, respectively. The results showed that zirconium doping significantly reduced the apparent activation energy of the catalyst. According to existing pieces of literature, the lower the activation energy of the catalyst, the higher the catalytic SCR activity (Wu et al., 2020).

**FIGURE 10:** Arrhenius diagram of Mn_6_Zr_1_ and Mn_6_Zr_0.3_Co_0.7_ catalysts.

The article "Effect of Bimetal Element Doping on the Low-Temperature Activity of Manganese-Based Catalysts for NH3-SCR" was retracted in 2023. Reason: duplicate publication.

## Analysis of Catalytic Mechanism

The Mn_6_Zr_0.3_Co_0.7_ catalyst prepared doping zirconium and cobalt into the MnO_x_ shows excellent denitrification ability and has a wide temperature window. The Mn_6_Zr_0.3_Co_0.7_ catalyst has a large specific surface area and abundant mesopores, which provides a convenient opportunity for gas adsorption and diffusion, thus improving the denitrification activity of the catalyst. Amorphous MnO_x_, ZrO_2,_ and CoO_x_ are formed on the surface of the Mn_6_Zr_0.3_Co_0.7_ catalyst, which are the main active oxides on the surface of the catalyst, promoting SCR denitration of the catalyst. The elemental valence states on the surface of the Mn_6_Zr_0.3_Co_0.7_ catalyst were characterized by XPS technology. The Mn^4+^, O_α,_ and Co^3+^ species on the surface of the Mn_6_Zr_0.3_Co_0.7_ catalyst were increased. Mn^4+^ is considered to be one of the best low-temperature denitrification species. Adsorbed oxygen O_α_ has excellent oxygen mobility, which enables the rapid oxidation of NO to NO_2_, resulting in a Fast SCR reaction. Co^3+^ can promote the oxygen reduction performance of the catalyst. The surface acidity of the Mn_6_Zr_0.3_Co_0.7_ catalyst was enhanced, which made it easier for the catalyst to adsorb NH_3_ and activate or decompose NH_3_ on its surface. At the same time, the reduction experiment of the Mn_6_Zr_0.3_Co_0.7_ catalyst shows that the reduction temperature of the Mn_6_Zr_0.3_Co_0.7_ catalyst decreases, which corresponds to the excellent denitrification activity of the catalyst at low temperature. In addition, the Lewis and Brønsted acid sites were found on the surface of the Mn_6_Zr_0.3_Co_0.7_ catalysts.

The common NO removal process is divided into two steps: NO reacts with O_2_ to form N_x_O_y_, which is further reduced to N_2_ by adsorbed NH_3_. The former is closely related to reactive oxygen species, including lattice oxygen and adsorbed oxygen, while the latter participates in the cleavage of the N-H bond in NH_3_ adsorbed on the Lewis acid site. Migration of H or NH_3_ combines with a surface hydroxyl group to form NH_4_^+^ adsorbed on the Bronsted acid site. They can form intermediates NH_4_NO_2_, NH_4_NO_3_, and NH_2_NO. Finally, these intermediates decompose into N_2_ and H_2_O. The Mn_6_Zr_0.3_Co_0.7_ catalyst exhibits superior NH_3_-SCR denitrification capacity, which is mainly attributed to the excellent physicochemical properties of the catalyst. Combining the results with references (Jiang et al., 2021; Kang et al., 2021), the reaction path of the Mn_6_Zr_0.3_Co_0.7_ catalyst can be described by E-R and L-H mechanisms. The whole reaction process is shown in Figure 11.

The article "Effect of Bimetal Element Doping on the Low-Temperature Activity of Manganese-Based Catalysts for NH3-SCR" was retracted in 2023. Reason: duplicate publication.

**FIGURE 11:** Reaction mechanism of the Mn_6_Zr_0.3_Co_0.7_ catalyst.

## Conclusion

In this study, a series of Mn_6_Zr_0.3_Co_0.7_ catalysts were prepared by doping of cobalt into the Mn_6_Zr_1_ catalyst. The catalytic performance of the doped catalyst has been significantly improved in low-temperature denitrification performance, sulfur resistance, and water resistance. To be specific, the NO_x_ conversion of the Mn_6_Zr_0.3_Co_0.7_ catalyst is above 90% in the reaction temperature range of 100–275°C, and the best NO_x_ conversion is up to 99%. Under 200 ppm SO_2_, the NO_x_ conversion still remains above 90%. Under 5Vol% H_2_O, the NO_x_ conversion basically remains at about 95%. According to the analysis of the characterization results, the Mn_6_Zr_0.3_Co_0.7_ catalyst has a large specific surface area, pore size, pore volume, and strong redox performance, which are the main reasons for the excellent catalytic activity.

## Data Availability

The raw data supporting the conclusions of this article will be made available by the authors, without undue reservation.

## References

[B1] AliS.ChenL.YuanF.LiR.ZhangT.BakhtiarS. u. H. (2017). Synergistic Effect between Copper and Cerium on the Performance of Cu X -Ce 0.5-x -Zr 0.5 ( X = 0.1-0.5) Oxides Catalysts for Selective Catalytic Reduction of NO with Ammonia. Appl. Catal. B Environ. 210, 223–234. 10.1016/j.apcatb.2017.03.065

[B2] AzalimS.FrancoM.BrahmiR.GiraudonJ.-M.LamonierJ.-F. (2011). Removal of Oxygenated Volatile Organic Compounds by Catalytic Oxidation over Zr-Ce-Mn Catalysts. J. Hazard. Mater. 188, 422–427. 10.1016/j.jhazmat.2011.01.135 21354699

[B3] BoningariT.EttireddyP. R.SomogyvariA.LiuY.VorontsovA.McDonaldC. A. (2015). Influence of Elevated Surface Texture Hydrated Titania on Ce-Doped Mn/TiO2 Catalysts for the Low-Temperature SCR of NO under Oxygen-Rich Conditions. J. Catal. 325, 145–155. 10.1016/j.jcat.2015.03.002

[B4] ChenJ.FuP.LvD.ChenY.FanM.WuJ. (2021). Unusual Positive Effect of SO2 on Mn-Ce Mixed-Oxide Catalyst for the SCR Reaction of NOx with NH3. Chem. Eng. J. 407, 127071–127110. 10.1016/j.cej.2020.127071

[B5] ChenQ.-l.GuoR.-t.WangQ.-s.PanW.-g.WangW.-h.YangN.-z. (2016). The Catalytic Performance of Mn/TiWO Catalyst for Selective Catalytic Reduction of NO with NH3. Fuel 181, 852–858. 10.1016/j.fuel.2016.05.045

[B6] ChenQ.-l.GuoR.-t.WangQ.-s.PanW.-g.WangW.-h.YangN.-z. (2016). The Catalytic Performance of Mn/TiWO Catalyst for Selective Catalytic Reduction of NO with NH3. Fuel 181, 852–858. 10.1016/j.fuel.2016.05.045

[B7] ChenS.VasiliadesM. A.YanQ.YangG.DuX.ZhangC. (2020). Remarkable N2-Selectivity Enhancement of Practical NH3-SCR over Co0.5Mn1Fe0.25Al0.75Ox-LDO: The Role of Co Investigated by Transient Kinetic and DFT Mechanistic Studies. Appl. Catal. B Environ. 277, 119186–119219. 10.1016/j.apcatb.2020.119186

The article "Effect of Bimetal Element Doping on the Low-Temperature Activity of Manganese-Based Catalysts for NH3-SCR" was retracted in 2023. Reason: duplicate publication.

[B8] FanZ.ShiJ.-W.GaoC.GaoG.WangB.WangY. (2018). Gd-modified MnOx for the Selective Catalytic Reduction of NO by NH3: The Promoting Effect of Gd on the Catalytic Performance and Sulfur Resistance. Chem. Eng. J. 348, 820–830. 10.1016/j.cej.2018.05.038

[B9] FangC.ZhangD.CaiS.ZhangL.HuangL.LiH. (2013). Low-temperature Selective Catalytic Reduction of NO with NH3 over Nanoflaky MnOx on Carbon Nanotubes *In Situ* Prepared via a Chemical Bath Deposition Route. Nanoscale 5, 9199–9207. 10.1039/c3nr02631k 23928911

[B10] FangN.GuoJ.ShuS.LuoH.ChuY.LiJ. (2017). Enhancement of Low-Temperature Activity and Sulfur Resistance of Fe 0.3 Mn 0.5 Zr 0.2 Catalyst for NO Removal by NH 3 -SCR. Chem. Eng. J. 325, 114–123. 10.1016/j.cej.2017.05.053

[B11] FangN.GuoJ.ShuS.LuoH.LiJ.ChuY. (2018). Effect of Calcination Temperature on Low-Temperature NH3-SCR Activity and the Resistance of SO2 with or without H2O over Fe-Mn-Zr Catalyst. J. Taiwan Inst. Chem. Eng. 93, 277–288. 10.1016/j.jtice.2018.07.027

[B12] FranceL. J.YangQ.LiW.ChenZ.GuangJ.GuoD. (2017). Ceria Modified FeMnO -Enhanced Performance and Sulphur Resistance for Low-Temperature SCR of NOx. Appl. Catal. B Environ. 206, 203–215. 10.1016/j.apcatb.2017.01.019

[B13] GaoF.TangX.YiH.ZhaoS.WangJ.ShiY. (2018). Novel Co- or Ni-Mn Binary Oxide Catalysts with Hydroxyl Groups for NH3-SCR of NOx at Low Temperature. Appl. Surf. Sci. 443, 103–113. 10.1016/j.apsusc.2018.02.151

[B14] GaoF.WalterE. D.KollarM.WangY.SzanyiJ.PedenC. H. F. (2014). Understanding Ammonia Selective Catalytic Reduction Kinetics over Cu/SSZ-13 from Motion of the Cu Ions. J. Catal. 319, 1–14. 10.1016/j.jcat.2014.08.010

[B15] GeZ.ShenY.GuS. (2022). High-temperature Selective Catalytic Reduction of NO with NH3: Optimization of ZrO2 and WO3 Complex Oxides. Fuel 310, 122261–122268. 10.1016/j.fuel.2021.122261

[B16] GongP.XieJ.FangD.HeF.LiF.QiK. (2020). Enhancement of the NH3-SCR Property of Ce-Zr-Ti by Surface and Structure Modification with P. Appl. Surf. Sci. 505, 144641–144649. 10.1016/j.apsusc.2019.144641

[B17] GuoM.LiuQ.LiuC.WangX.BiY.FanB. (2021). Rational Design of Novel CrZrO Catalysts for Efficient Low Temperature SCR of NO. Chem. Eng. J. 413, 127554. 10.1016/j.cej.2020.127554

[B18] HanS.ChengJ.YeQ.ChengS.KangT.DaiH. (2019). Ce Doping to Cu-SAPO-18: Enhanced Catalytic Performance for the NH3-SCR of NO in Simulated Diesel Exhaust. Microporous Mesoporous Mater. 276, 133–146. 10.1016/j.micromeso.2018.09.027

[B19] HuG.YangJ.TianY.KongB.LiuQ.RenS. (2018). Effect of Ce Doping on the Resistance of Na over V2O5-WO3/TiO2 SCR Catalysts. Mater. Res. Bull. 104, 112–118. 10.1016/j.materresbull.2018.04.009

The article "Effect of Bimetal Element Doping on the Low-Temperature Activity of Manganese-Based Catalysts for NH3-SCR" was retracted in 2023. Reason: duplicate publication.

[B20] HuH.CaiS.LiH.HuangL.ShiL.ZhangD. (2015). *In Situ* DRIFTs Investigation of the Low-Temperature Reaction Mechanism over Mn-Doped Co3O4 for the Selective Catalytic Reduction of NOx with NH3. J. Phys. Chem. C 119, 22924–22933. 10.1021/acs.jpcc.5b06057

[B21] HuX.ShiQ.ZhangH.WangP.ZhanS.LiY. (2017). NH 3 -SCR Performance Improvement over Mo Modified Mo(x)-MnO X Nanorods at Low Temperatures. Catal. Today 297, 17–26. 10.1016/j.cattod.2017.06.015

[B22] HuangX.DongF.ZhangG.GuoY.TangZ. (2021). A Strategy for Constructing Highly Efficient Yolk-Shell Ce@Mn@TiOx Catalyst with Dual Active Sites for Low-Temperature Selective Catalytic Reduction of NO with NH3. Chem. Eng. J. 419, 129572–129613. 10.1016/j.cej.2021.129572

[B23] JiaB.GuoJ.LuoH.ShuS.FangN.LiJ. (2018). Study of NO Removal and Resistance to SO2 and H2O of MnO /TiO2, MnO /ZrO2 and MnO /ZrO2-TiO2. Appl. Catal. A General:Gen 553, 82–90. 10.1016/j.apcata.2017.12.016

[B24] JiaB.GuoJ.ShuS.FangN.LiJ.ChuY. (2017). Effects of Different Zr/Ti Ratios on NH3-SCR over MnO /Zr Ti1-O2: Characterization and Reaction Mechanism. Mol. Catal. 443, 25–37. 10.1016/j.mcat.2017.09.019

[B25] JiangH.GuanB.PengX.ZhanR.LinH.HuangZ. (2020). Influence of Synthesis Method on Catalytic Properties and Hydrothermal Stability of Cu/SSZ-13 for NH3-SCR Reaction. Chem. Eng. J. 379, 122358–122415. 10.1016/j.cej.2019.122358

[B26] JiangS. J.SongS. Q. (2013). Enhancing the Performance of Co3O4/CNTs for the Catalytic Combustion of Toluene by Tuning the Surface Structures of CNTs. Appl. Catal. B:Environ 140, 1–8. 10.1016/j.apcatb.2013.03.040

[B27] JiangY.LiuT.LaiC.YangZ.LinR.WangX. (2021). Deactivation of CeO2-TiO2 Catalyst by K2SO4 for NH3-SCR: An Experimental and DFT Study. Appl. Surf. Sci. 547, 149196–149210. 10.1016/j.apsusc.2021.149196

[B28] JinQ.ShenY.MeiC.ZhangY.ZengY. (2022). Catalytic Removal of NO and Dioxins over W-Zr-Ox/Ti-Ce-Mn-Ox from Flue Gas: Performance and Mechanism Study. Catal. Today 388-389, 372–382. 10.1016/j.cattod.2020.05.061

[B29] KangK.YaoX.HuangY.CaoJ.RongJ.ZhaoW. (2021). Insights into the Co-doping Effect of Fe3+ and Zr4+ on the Anti-K Performance of CeTiOx Catalyst for NH3-SCR Reaction. J. Hazard. Mater. 416, 125821–125913. 10.1016/j.jhazmat.2021.125821 33866288

[B30] KantchevaM.CayirtepeI.NaydenovA.IvanovG. (2011). FT-IR Spectroscopic Investigation of the Effect of SO2 on the SCR of NOx with Propene over ZrO2-Nb2O5 Catalyst. Catal. Today 176, 437–440. 10.1016/j.cattod.2010.10.072

[B31] KwonD. W.ParkK. H.HongS. C. (2016). Enhancement of SCR Activity and SO 2 Resistance on VO X /TiO 2 Catalyst by Addition of Molybdenum. Chem. Eng. J. 284, 315–324. 10.1016/j.cej.2015.08.152

The article "Effect of Bimetal Element Doping on the Low-Temperature Activity of Manganese-Based Catalysts for NH3-SCR" was retracted in 2023. Reason: duplicate publication.

[B32] LamonierJ.-F.BoutoundouA.-B.GennequinC.Pérez-ZuritaM. J.SiffertS.AboukaisA. (2007). Catalytic Removal of Toluene in Air over Co-mn-al Nano-Oxides Synthesized by Hydrotalcite Route. Catal. Lett. 118, 165–172. 10.1007/s10562-007-9196-4

[B33] LiuY.GuT.WengX.WangY.WuZ.WangH. (2012). DRIFT Studies on the Selectivity Promotion Mechanism of Ca-Modified Ce-Mn/TiO2 Catalysts for Low-Temperature NO Reduction with NH3. J. Phys. Chem. C 116, 16582–16592. 10.1021/jp304390e

[B34] MengB.ZhaoZ.WangX.LiangJ.QiuJ. (2013). Selective Catalytic Reduction of Nitrogen Oxides by Ammonia over Co3O4 Nanocrystals with Different Shapes. Appl. Catal. B Environ. 129, 491–500. 10.1016/j.apcatb.2012.09.040

[B35] PanY.ShenB.LiuL.YaoY.GaoH.LiangC. (2020). Develop High Efficient of NH3-SCR Catalysts with Wide Temperature Range by Ball-Milled Method. Fuel 282, 118834–118914. 10.1016/j.fuel.2020.118834

[B36] ShiA.WangX.YuT.ShenM. (2011). The Effect of Zirconia Additive on the Activity and Structure Stability of V2O5/WO3-TiO2 Ammonia SCR Catalysts. Appl. Catal. B Environ. 106, 359–369. 10.1016/j.apcatb.2011.05.040

[B37] SunX.GuoR.-t.LiuJ.FuZ.-g.LiuS.-w.PanW.-g. (2018). The Enhanced SCR Performance of Mn/TiO2 Catalyst by Mo Modification: Identification of the Promotion Mechanism. Int. J. Hydrogen Energy 43, 16038–16048. 10.1016/j.ijhydene.2018.07.057

[B38] TangX.HaoJ.XuW.LiJ. (2007). Low Temperature Selective Catalytic Reduction of NO with NH3 over Amorphous MnO Catalysts Prepared by Three Methods. Catal. Commun. 8, 329–334. 10.1016/j.catcom.2006.06.025

[B39] TangX.WangC.GaoF.MaY.YiH.ZhaoS. (2020). Effect of Hierarchical Element Doping on the Low-Temperature Activity of Manganese-Based Catalysts for NH3-SCR. J. Environ. Chem. Eng. 8, 104399–104410. 10.1016/j.jece.2020.104399

[B40] ThirupathiB.SmirniotisP. G. (2011). Co-doping a Metal (Cr, Fe, Co, Ni, Cu, Zn, Ce, and Zr) on Mn/TiO2 Catalyst and its Effect on the Selective Reduction of NO with NH3 at Low-Temperatures. Appl. Catal. B Environ. 110, 195–206. 10.1016/j.apcatb.2011.09.001

[B41] WangR.HaoZ.LiY.LiuG.ZhangH.WangH. (2019). Relationship between Structure and Performance of a Novel Highly Dispersed MnOx on Co-al Layered Double Oxide for Low Temperature NH3-SCR. Appl. Catal. B Environ. 258, 117983–117989. 10.1016/j.apcatb.2019.117983

[B42] WangX.WuS.ZouW.YuS.GuiK.DongL. (2016). Fe-Mn/Al 2 O 3 Catalysts for Low Temperature Selective Catalytic Reduction of NO with NH 3. Chin. J. Catal. 37, 1314–1323. 10.1016/S1872-2067(15)61115-9

[B43] WuR.LiL.ZhangN.HeJ.SongL.ZhangG. (2021). Enhancement of Low-Temperature NH3-SCR Catalytic Activity and H2O & SO2 Resistance over Commercial V2O5-MoO3/TiO2 Catalyst by High Shear-Induced Doping of Expanded Graphite. Catal. Today 376, 302–310. 10.1016/j.cattod.2020.04.051

The article "Effect of Bimetal Element Doping on the Low-Temperature Activity of Manganese-Based Catalysts for NH3-SCR" was retracted in 2023. Reason: duplicate publication.

[B44] WuX.MengH.DuY.LiuJ.HouB.XieX. (2020). Insight into Cu2O/CuO Collaboration in the Selective Catalytic Reduction of NO with NH3: Enhanced Activity and Synergistic Mechanism. J. Catal. 384, 72–87. 10.1016/j.jcat.2020.01.025

[B45] XiongS.PengY.WangD.HuangN.ZhangQ.YangS. (2020). The Role of the Cu Dopant on a Mn3O4 Spinel SCR Catalyst: Improvement of Low-Temperature Activity and Sulfur Resistance. Chem. Eng. J. 387, 124090–124112. 10.1016/j.cej.2020.124090

[B46] ZhaiG.HanZ.WuX.DuH.GaoY.YangS. (2021). Pr-modified MnO Catalysts for Selective Reduction of NO with NH3 at Low Temperature. J. Taiwan Inst. Chem. Eng. 125, 132–140. 10.1016/j.jtice.2021.06.008

[B47] ZhangK.YuF.ZhuM.DanJ.WangX.ZhangJ. (2018). Enhanced Low Temperature NO Reduction Performance via MnOx-Fe2O3/Vermiculite Monolithic Honeycomb Catalysts. Catalysts 8, 100–115. 10.3390/catal8030100

[B48] ZhangL.ShiL.HuangL.ZhangJ.GaoR.ZhangD. (2014). Rational Design of High-Performance DeNOx Catalysts Based on MnxCo3-xO4 Nanocages Derived from Metal-Organic Frameworks. ACS Catal. 4, 1753–1763. 10.1021/cs401185c

[B49] ZhangY.ZhengY.WangX.LuX. (2015). Preparation of Mn-FeOx/CNTs Catalysts by Redox Co-precipitation and Application in Low-Temperature NO Reduction with NH3. Catal. Commun. 62, 57–61. 10.1016/j.catcom.2014.12.023

[B50] ZhangZ.LiR.WangM.LiY.TongY.YangP. (2021). Two Steps Synthesis of CeTiOx Oxides Nanotube Catalyst: Enhanced Activity, Resistance of SO2 and H2O for Low Temperature NH3-SCR of NOx. Appl. Catal. B Environ. 282, 119542–119612. 10.1016/j.apcatb.2020.119542

[B51] ZhouX.DanJ.ZhangJ.YangS.ShiL.WangJ. (2019). Two-dimensional MnAl Mixed-Metal Oxide Nanosheets Prepared via a High-Shear-Mixer-Facilitated Coprecipitation Method for Enhanced Selective Catalytic Reduction of NO with NH3. Chem. Eng. Process. - Process Intensif. 145, 107664–107669. 10.1016/j.cep.2019.107664

